RETRACTED

# Inhibitor 9 Combined With Androgen Deprivation Therapy or Chemotherapy Delays the Malignant Behavior of Castration-Resistant Prostate Cancer Through K-Ras/PLCε/PKCε Signaling Pathway

**DOI:** 10.3389/fonc.2020.00075

**Published:** 2020-02-25

**Authors:** Jiayu Liu, Yongbo Zheng, Yingying Gao, Zhen Quan, Bo Qiao, Luo Li, Ting Li, Limei Duan, Jinxiao Yang, Chunli Luo, Xiaohou Wu

**Affiliations:** ^1^Department of Urology, The First Affiliated Hospital of Chongqing Medical University, Chongqing, China; ^2^Department of Laboratory Diagnosis, Chongqing Medical University, Chongqing, China; ^3^Department of Laboratory Diagnosis, Clinical Medical College, Jiamusi University, Heilongjiang, China; ^4^Department of Orthopaedics, The First Affiliated Hospital of Chongqing Medical University, Chongqing, China; ^5^Department of Laboratory Diagnosis, Chongqing Public Health Medical Treatment Center, Chongqing, China

**Keywords:** KRAS mutation G12C, inhibitor 9, castration-resistant prostate cancer, drug resistance, metastasis

## Abstract

Castration-resistant prostate cancer (CRPC) is a progressed stage of prostate cancer, which requires better understanding of the mechanisms and remains an unmet clinical need. As a common oncogene, K-Ras is associated with malignant behavior in different types of tumors but its role in CRPC is unknown. The present study aims to find the mechanism of K-Ras in CRPC and whether it can be used as a crucial molecule for the treatment of CRPC. For this purpose, tissue samples from primary prostate cancer (PPC) and CRPC patients were analyzed by immunohistochemistry and the data showed that K-Ras was elevated in CRPC. More importantly, higher K-Ras expression was related to a shorter recurrence-free survival time in patients with CRPC. In addition, K-Ras promoted the invasion, migration, and drug resistance of CRPC cells by activation of PLCε/PKCε signaling pathway. Meanwhile, the inhibitor of K-RasG12C mutants was able to inhibit malignant behavior of CRPC cells *in vitro* and *in vivo*. Inhibitors of K-RasG12C mutants have entered clinical trials. Taken together, the study shows that K-Ras may activate PKCε through PLCε, resulting in the alterations of malignant behavior of CRPC. Inhibitor 9, an inhibitor of the K-RasG12C mutant, has a strong anti-tumor effect in CRPC, which potentially suggests that inhibitors of this nature may serve as a promising treatment for CRPC.

## Introduction

Prostate cancer is one of the most common types of male urinary tumors and the fifth cause of cancer-related death in men (1–4), and its incidence in China is increasing annually (5, 6). Previous studies reported that the pathogenesis of prostate cancer was related to the androgen receptor (AR) (7–10). After surgery, patients are often treated with androgen deprivation therapy (ADT), generally consisting of new AR inhibitor drugs such as enzalutamide and abiraterone (11–13). These treatments are always initially successful in patients, but almost all tumors will eventually develop resistance against these drugs, namely, CRPC. Chemotherapy drugs are currently the preferred treatment for patients with CRPC. However, these prostate cancers will always become dually resistant against both the ADT and chemotherapy drugs in just a few months (1, 14–16), which can have adverse effects on the patient's survival. Thus, new treatments for refractory prostate cancer are urgently needed.

RETRACTED

The RAS genes are believed to be one of the most common oncogene families in human tumors and mutated in nearly one-third of human cancers (17–19). Recent studies reported a 12th codon mutation as the most common one in this gene (20–22). Reports have also demonstrated that K-Ras mutation activation is related to tumor drug resistance, metastasis, and even increased mortality (23–26). Our previous studies have shown that K-Ras expression is up-regulated in CRPC cells and is related to invasion, but the underlying mechanism is unknown. Meanwhile, it has been shown that PKCε is associated with drug resistance in tumors (27). It is worth noting that reduced PKCε expression has been reported in normal or benign prostatic epithelial cells and androgen-dependent prostate cancer cells (28, 29), with high expression reported in CRPC cells (30, 31). Thus, it is worth exploring whether PKCε activation is related to prostate cancer progression. In previous studies from our research group and others, PLCε has been suggested to play an important role in human malignancies (32–36). In addition, PLCε as a subtype of the PLC family has a unique structure: RA domain may directly bind to the RAS gene family and the common structures of the PLC family: EF, X, and F can activate DAG/CA2+ to activate PKC (37). Therefore, whether PLCε can be regulated by the Ras family through the RA structure, and whether it can regulate the activation of PKC kinase through a second messenger in CRPC is currently unknown.

The aim of our study is to explore whether K-Ras is capable of binding and activating PLCε. Subsequently, activated PLCε could directly interact with PKCε, thereby regulating the malignant behavior of CRPC. In addition, whether inhibitor 9, an inhibitor of K-RasG12C mutants, can delay this lethal progression remains to be determined.

For this purpose, we assessed the expression of K-Ras, PLCε, and PKCε in CRPC and PPC tissues by immunohistochemistry and different types of cell lines *in vitro and in vivo* to explore treatment strategies. Collectively, the present study suggests that inhibiting K-Ras can significantly delay the malignant behavior of CRPC cells and that the combined therapy of inhibitor 9 and ADT with or without chemotherapy may supply a new treatment strategy for patients with refractory prostate cancer.

RETRACTED

## Materials and Methods

### Patients and Tissue Samples

Tissue samples from 50 PPC patients and 41 CRPC patients were collected at the First Affiliated Hospital of Chongqing Medical University (Chongqing, China) between January 2010 and July 2019. Histological examination confirmed that all tissue samples were positive for prostate adenocarcinoma. Informed consent was acquired for all patients. In our study, CRPC patients were defined in accordance with the guidelines of the European Association of Urology (EU) (38). Here, we retrospectively analyzed patient's age, prostate-specific antigen (PSA) levels, metastasis, and drug resistance. The study was approved by the Ethics Committee of Chongqing Medical University and conducted according to the principles of the Helsinki Declaration.

### Immunohistochemistry

Tumor tissues were embedded in 10% paraformaldehyde for 12 h at 24°C and cut into paraffin sections. Immunohistochemical staining was performed by standard immunoperoxidase-based visualization. All tissues were incubated with antibodies [K-Ras, PLCε, and PKCε (Santa Cruz)] overnight at 4°C. Secondary antibody was incubated for 1 h at around 37°C. Target expression was confirmed by staining with diamino phenylaniline for 5 min followed by counterstaining with hematoxylin for 5 min at 25°C. The intensity of tissue staining was analyzed using IMAGE J software and the relevant results were statistically analyzed.

### Cell Culture and Treatment

The LNCaP cell line was obtained from American type culture specimens. To induce resistance, LNCaP cells were cultured in drug resistance media (39–41). Cells exhibiting bicalutamide resistance were named R-Bica cells and LNCaP cells resistant to bicalutamide and docetaxel were named R-B+D cells as previously described (41).

### Transduction

A total of 1 × 10^5^ cells were cultured in 6-well plates and passaged every 2 days. When the cells reached 40–60% confluence, they were transduced with either 3 μg of K-Ras-silenced lentivirus (sh-K-Ras) (#1, CCTTGACGATACAGCTAATTC; #2, GACGAATATGATCCAACAATA; #3, GAGGGCTTTCTTTGTGTATTT) or negative control. Infection was allowed to continue for 8 h, after which cells were added to the basal medium supplemented with 1 μg/ml puromycin. These cells were used for RNA extraction after 48 h and protein extraction after 72 h. For the knockdown of PLCε [GGTTCTCTCCTAGAAGCAACC, our previously study had verified (35)], PKCε (#1, CCCTTCAAACCACGCATTAAA; #2, CTGCATGTTCAGGCATATTAT; #3, ATATGCTGTGAAGGTCTTAAA) or the method of K-RasG12C mutation lentivirus was the same.

RETRACTED

### RNA Extraction and RT-PCR

Total RNA was extracted by TRIzol reagent. For each cell line, 1 μg of RNA was reverse transcribed to synthesize cDNA by the Prime Script^TM^ RT reagent kit according to the manufacturer's instructions. The mRNA levels in all cell lines were analyzed by qRT-PCR by the PremixEx Taq^TM^ II kit and a CFX 96-well RT-PCR Detection System. K-Ras, PLCε, PKCε, K-RasG12C, VEGF, MPP2, and MMP9 related the expression of mRNA levels and were calculated by the comparative 2.ΔΔCq method (42) using β-actin as the calibrator. mRNA analysis was performed in triplicate. Primers used for gene amplifications are listed below:

K-Ras, Forward: ATTTTGTGGACGAATATGATCCAAC
Reverse: GCTGTGTCGAGAATATCCAAGAGAC
K-RasG12C, Forward: TGTGGTAGTTGGAGCTGGTG
Reverse: TGACCTGCTGTGTCGAGAAT
PLCε, Forward: GCAACTACAACGCTGTCATGGAG
Reverse: CCTCATGGTCTCAATATCAGACTGG
PKCε, Forward: AAACACCCTTATCTAACCCAACTCT
Reverse: CATATTCCATGACGAAGAAGAGC
VEGF, Forward: TTGCTGCTCTACCTCCAC
Reverse: AATGCTTTCTCCGCTCTG
MMP2, Forward: GATGCCGCCTTTAACTGG
Reverse: TCAGCAGCCTAGCCAGTCG
MMP9, Forward: GAGGAATACCTGTACCGCTATG
Reverse: CAAACCGAGTTGGAACCAC
β-actin, Forward: TGACGTGGACAT CCGCAAAG
Reverse: CTGGAAGGTGGACAG CGAGG

### Western Blot Assay

Total protein from cells and tissue samples was extracted as previously described (43). Membrane and plasma proteins were extracted using the relevant extraction kits. The concentration of protein was detected using BCA protein assay. Isolated proteins were analyzed by sodium dodecyl sulfate–polyacrylamide gel electrophoresis. After protein was separated, it was transferred to a polyvinylidene difluoride membrane. The membrane was incubated overnight with the following primary antibodies: K-Ras, PLCε, and PKCε (Santa Cruz); and VEGF, MMP2, MMP9, and β-actin (Cell Signaling Technology). Next, the membrane was incubated with secondary antibody for 2 h, and finally visualized by Enhanced Chemiluminescence (41, 44). Image-Pro Plus 6.0 software was used for detecting protein band intensity.

### Co-immunoprecipitation

Total protein extraction was performed as previously described. Total lysates were divided into “input” groups (for detecting the expression of K-Ras and PLCε), IgG groups, and “IP” groups. The “IP” group was treated with anti-K-Ras, and the “IgG” group was incubated with only the lgG antibodies overnight at 4° and then immunoprecipitate using Protein A/G Plus-Agarose. Beads were washed three times and boiled in SDS sample buffer and then separated using SDS-PAGE and following the Western blot assay. Groups for PLCε and PKCε were treated similarly.

RETRACTED

### Cellular Analysis Assay

Approximately 2,000 cells per well were placed in 96-well-plates and cultured for 12 h at 37°C until they reached confluence. Cells were then cultured under different treatment and concentration conditions in each of the five replicate wells for 24–72 h. A CCK-8 kit was used to evaluate cell health. Reagents were added into each well for 2 h at 37°C, and then the absorbance was analyzed at 450 nm on a microplate reader. In this assay, we measured the growth of cells over 96 h and calculated the ratio of bicalutamide or bicalutamide and docetaxel in R-Bica or R-B+D cells under varying conditions.

### Transwell Invasion and Wound-Healing Assays

In the Transwell invasion assay, 1,000 cells were plated per well on a matrix-coated membrane in the upper chamber of the Transwell apparatus and cultured with serum-free medium. After incubating for 24 h at 37°C, the cells were stained with 4% paraformaldehyde for 20 min. Then, cells were stained with 0.1% crystal violet for 10 min at 25°C. Finally, cells were counted using a fluorescence microscope. The average from five separate fields of view was then determined.

In the wound-healing assays, 5 × 10^4^ cells were cultured in 6-well plates per well and seeded with serum-free medium at 37°C for 24 h. The cell monolayer was wounded with a 200-μl pipette to form gap, washed with PBS, and cultured at 37°C for 1 day. Images were taken using an inverted microscope at various time points.

### Colony Formation Assay

A total of 400 cells were cultured in 6-well plates each well and the medium was refreshed every 3 days. After 2 weeks, cells were stained with 0.05% crystal violet for 20 min at 25°C. Colony numbers were counted using bright-field microscopy.

### Animal Study

The animal experiments were approved by the Ethics Committee of Chongqing Medical University. To develop a metastasis model, 3 × 10^8^ R-Bica and R-B+D cells transduced with lentivirus expressing firefly luciferase were injected via the tail vein to nude mice. We detected tumor metastasis on an IVIS Lumina II with imaging each week. To facilitate this, 3 mg of D-luciferin was injected via the tail vein of isoflurane-anesthetized mice. The intensity of the fluorescence is expressed using radiance, calculated as p/s/cm^2^/sr.

To create bone invasion models or the subcutaneous tumor, 3 × 10^8^ R-Bica or R-B+D cells were injected into left tibia of nude mice or the right flank and xenograft tumors were monitored every 5 days with its volume calculated as 1/2 × length × width^2^. Bone invasion was monitored using weekly X-rays and finally stained by hematoxylin and eosin (HE).

RETRACTED

In all three animal models, we divided the nude mice into four groups: R-Bica (injected bicalutamide and PBS via tail vein) and R-B+D (injected bicalutamide, docetaxel, and PBS via tail vein) were the control groups, and R-Bica inhibitor 9 (injected bicalutamide and inhibitor 9 via tail vein) and R-B+D inhibitor 9 (injected bicalutamide, docetaxel, and inhibitor 9 via tail vein) were the experimental groups with a total of five mice per group. The dose of the inhibitor 9, bicalutamide, docetaxel, and PBS was 10 mg/kg. All treatments consisted of 5 days on and 2 days off for a total of 42 days.

### Statistical Analysis

The experiments of this study were repeated at least three times, and statistical significance tests were undertaken using the statistical analysis software GraphPad Prism version 5 and SPSS version 21.0. Significant differences were analyzed among groups by one-way analysis of variance (ANOVA), the Student's *t* test, and two-way ANOVA. Multiple comparison corrections were performed using the Bonferroni adjustment, and survival analysis was done by the Kaplan-Meier method. Other data were analyzed using the Mann–Whitney test, Spearman correlation, and Chi-square test. The Student–Newman–Keuls test was used for *post-hoc* testing. Multiple comparisons were assessed using one-way ANOVA. Results were considered to be statistically significant when *P* < 0.05.

## Results

### Increased K-Ras Is Associated With Increased Expression of PLCε and PKCε in CRPC Tissues

The demographics and clinical characteristics of participants in the K-Ras study are provided in Table 1. A total of 50 primary prostate cancer and 41 CRPC samples were collected (Table 1) and the data showed that 65% of CRPC patients and only 52% of PPC patients exhibited high levels of K-Ras expression. Among all the clinical parameters, bone and visceral metastases were the only parameters that positively correlated with the expression of K-Ras (*P* = 0.009, *P* = 0.046 in CRPC samples and *P* = 0.01, *P* = 0.018 in PPC samples), suggesting that K-Ras overexpression may promote bone and visceral metastases. In CRPC samples positive for bicalutamide resistance, 71% exhibited high K-Ras expression, and in samples with bicalutamide and docetaxel multidrug resistance, 59% had elevated K-Ras expression, indicating that elevated K-Ras may be positively related with drug resistance. IHC analysis revealed that expression of K-Ras, PLCε, and PKCε was significantly higher in CRPC tissues when compared to PPC tissues (*P* = 0.014, *P* = 0.007, *P* = 0.018) (Figures 1A,B). The expression level of K-Ras was positively correlated with the expression level of PLCε in CRPC patients (*r* = 0.40, *P* = 0.0084) and with PKCε (*r* = 0.42, *P* = 0.0065) (Figure 1C) using Spearman correlation analysis. To confirm these observations, we extracted the proteins from 13 CRPC samples for Western blot analysis. Western blot confirmed that the expression level of K-RAS in CRPC tissues was positively correlated with the expression of PLCε (*r* = 0.58, *P* = 0.04) and PKCε (*r* = 0.65, *P* = 0.02) (Figures 1E,F). In addition, the patients with lower K-Ras expression had a median recurrence-free survival (RFS) of 38 months (95% confidence interval, CI = 34–42 months), while CRPC patients with high K-Ras expression had a RFS of 27 months (95% CI = 25–30 months) using Kaplan–Meier survival analysis, revealing that K-Ras-positive CRPC patients were associated with a shorter RFS (*P* = 0.007, log rank test) (Figure 1D).

RETRACTED

**Table 1:** K-Ras associated with demographic and clinical characteristics of the patients in PPC or CRPC.

		**K-Ras**		
**Characteristics**	**Total**	**Positive (%)**	**Negative (%)**	
PPC	50	26 (52%)	24 (48%)	
CRPC	41	27 (65%)	14 (34%)	
Age of patients with PPC (years), *P* = 0.194^a^				
Median	63	64	63	
Quartiles 25–75	62–68	62–70	61–68	
Age of patients with CRPC (years)				*P* = 0.438^a^
Median	74	75	73	
Quartiles 25–75	70–80	71–80	69–79	
PSA of patients with PPC (μg/L)				*P* = 0.322^a^
Median	75.15	86.75	49.9	
Quartiles 25–75	42.45–501.02	42.35–532.9	42.4–490.42	
PSA of patients with CRPC (μg/L)				*P* = 0.165^a^
Median	25.6	32.55	20.7	
Quartiles 25–75	20.75–46.4	24.57–48.3	19.3–46.1	
Metastases in PPC				
Bone	20	15	5	***P* = 0.01^b^**
Visceral	17	13	4	***P*** **=** **0.018**^**b**^
Metastases in CRPC				
Bone	21	18	3	***P*** **=** **0.009**^**b**^
Visceral	19	16	3	***P*** **=** **0.046**^**b**^
Drug resistance (CRPC)				
Bicalutamide	24	17 (71%)	7 (29%)	
Bicalutamide+docetaxel	17	10 (59%)	7 (41%)	

a *Mann–Whitney test*.

b *Chi-square statistical significance numbers indicated in bold font*.

*PSA, prostate-specific antigen. IHC staining positive for K-Ras when the tissue staining is >23%*.

**Figure 1:** Expressions levels of K-Ras, PLCε, and PKCε in 50 PPC and 41 CRPC tumors. **(A)** K-Ras, PLCε, and PKCε expression in PPC and CRPC was detected by immunochemistry (magnification, ×200). **(B)** Image J was used to analyze the degree of tissue staining for K-Ras, PLCε, and PKCε in different tumor samples. **(C)** Correlation curve analysis for K-Ras staining scores vs. PLCε, PKCε staining scores in CRPC tissues. **(D)** The relationships of K-Ras with recurrence-free survival in CRPC patients. **(E)** Western blot was used to detect the protein expressions of K-Ras, PLCε, and PKCε in 13 CRPC tumor tissues; β-actin was used as a control. **(F)** Correlation curve analysis for the protein expressions of K-Ras vs. PLCε and PKCε in CRPC specimens. PLCε, phosphoinositide-specific phospholipase Cε. PKCε, protein kinase Cε. *p* < 0.05 was thought to be statistically significant.

RETRACTED

### Increased K-Ras Is Also Associated With Increased Metastasis and Invasion of CRPC Cells

To verify the underlying relationship between metastasis, invasion, and the expression of K-RAS, PLCε, and PKCε, we constructed two drug-resistant cell lines R-Bica and R-B+D cells. We used IC_50_ to evaluate the drug sensitivity of LNCaP cells and CRPC cell lines. The results showed that all CRPC cell lines had significantly higher IC_50_ values than the parental LNCaP cell line (Figure 2A). Then, we used Western blot and RT-qPCR to confirm K-Ras, PLCε, and PKCε protein, and mRNA expression in R-Bica and R-B+D cells was higher than those of LNCaP cells (Figure 2B). To demonstrate whether the high expression of K-Ras in drug-resistant cells is related to metastasis and invasion of CRPC cells, we constructed a lentivirus that knocked down the expression of K-Ras and used it to infect the resistant cell lines R-Bica and R-B+D. To silence K-Ras, CRPC cells were infected with three different lentiviral short hairpin (sh) RNAs specific for K-Ras(LV-sh-K-Ras#1, LV-sh-K-Ras #2, and LV-sh-K-Ras #3). LV-sh-K-Ras#1 markedly reduced the protein and mRNA expression of K-Ras (Figure 2C). Meanwhile, we analyzed factors related to metastasis, including VEGF, MMP2, and MMP9, using Western blot and RT-qPCR. The results suggested that the reduction in K-RAS expression down-regulated the expression of VEGF, MMP2, and MMP9 (Figure 2D). The Transwell and wound-healing assays consistently revealed that K-Ras silencing suppressed invasion and migration of CRPC cell lines (Figures 2E,F).

**Figure 2:** K-Ras, PLCε, and PKCε expression in LNCaP and CRPC cell lines and silencing K-Ras can suppress metastasis of CRPC cells. **(A)** IC_50_ was analyzed by cell counting kit-8 (CCK-8), and LNCaP and R-Bica cells were incubated with increasing concentrations of bicalutamide for 48 h; LNCaP and R-B+D cells were incubated with increasing concentrations of bicalutamide and docetaxel for 48 h. **(B)** The mRNA and protein levels of K-Ras, PLCε, and PKCε in LNCaP, R-Bica, and R-B+D cells were analyzed by Western blot analysis and qPCR. **(C)** CRPC cells were infected with lentiviral sh-K-Ras; Western blotting and qPCR detected the expression of K-Ras. **(D)** The expression of VEGF, MMP2, and MMP9 in CRPC cells was examined by Western blot and qPCR analysis. **(E,F)** The invasive and migratory capacities of CRPC cells were detected by Transwell and wound-healing assays. R-Bica cells, bicalutamide-resistant LNCap cells; R-E+D cells, sequential dual-resistant LNCap cells (bicalutamide-resistant and docetaxel-resistant LNCaP cells); sh, small hairpin; NC, negative control; shK-Ras, K-Ras knockdown. Data were presented as the means ± SD. **P < 0.01, ***P < 0.001; ns, no statistical significance.

RETRACTED

### Knockdown of K-Ras Suppressed the Proliferation of CRPC Cells and Partially Restores Drug Sensitivity

To verify the effect of targeting K-Ras on the drug resistance and proliferative capacity of CRPC cells, we examined the IC_50_ of bicalutamide in R-Bica and R-Bica cells with knocked-down K-Ras by CCK-8 method. We determined IC_50_ values for the parental R-Bica and the K-Ras knocked down line at 100.7 and 36.09 μM, respectively. In addition, the IC_50_ of bicalutamide and docetaxel in R-B+D and R-B+D knocked-down K-Ras lines were 113.3 and 45.49 μM, respectively (Figure 3A). The viability and proliferation of R-Bica, shK-Ras R-Bica, R-B+D, and shK-RasR-B+D cells were detected using CCK8 and clone formation assays. Here, we showed that knocking down K-Ras decreased proliferation abilities compared to the control group (Figures 3B,C). From these experiments, it can be concluded that knockdown of K-Ras can increase drug sensitivity and reduce proliferative ability of CRPC cells.

**Figure 3:** K-Ras knockdown suppressed cell proliferation in CRPC cells. **(A)** R-Bica cells were incubated with increasing concentrations of bicalutamide while R-B+D cells were incubated with increasing concentrations of bicalutamide, and bicalutamide and docetaxel for 48 h, and the IC_50_ of CRPC cells following treatment with LV-shK-Ras and LV-NC was determined by CCK-8 assay. **(B,C)** Proliferation efficiency of R-Bica and R-B+D cells was detected by colony forming assay and CCK-8 assay. *P < 0.05.

### Higher Expression of K-Ras Increased the Expression of PKCε Through Expression of PLCε in Membrane

As stated above, the mRNA and protein levels of K-Ras, PLCε, and PKCε in drug-resistant cell lines were higher than those of the LNCaP cells. Thereby, we hypothesized that K-Ras may regulate the membrane of PLCε and may be related with CRPC cell metastasis. To explore this concept, we knocked down K-Ras of CRPC cells, and mRNA and protein level expressions of PLCε and PKCε in K-Ras silenced CRPC cell lines had reduced when compared with the negative control group (Figure 4A). Studies reported that the main reason for activating K-Ras was the mutation of K-RAS (K-RASG12C) (22). We transfected the K-RASG12C mutant into our CRPC cells and the mRNA expression of K-RASG12C was elevated compared to the vector group (Figure 4B). In addition, the protein levels and mRNA of PKCε in K-RASG12C mutant CRPC cells, K-RASG12C mutant, and knocked-down PLCε CRPC cells were increased compared with the control group and the knocked-down PLCε group (Figure 4C) [our previous study had verified that one of the lentiviral shRNAs specific for PLCε can markedly reduce the mRNA and protein expression of PLCε we used in this study (35)]. Our previous studies showed that activation of PLCε was achieved by elevated membrane protein expression (45). So, we extracted membrane and cytoplasmic proteins in the PLCε knockdown and mutant-K-Ras CRPC cell lines. We concluded that mutant-K-Ras can activate PLCε in the membrane and thus PKCε (Figure 4D). To further elucidate the underlying mechanism of K-Ras in regulating PKCε through PLCε, we used co-immunoprecipitation, and the study revealed that K-Ras interacts with PLCε, and PLCε interacts with PKCε at the protein level (Figure 4E). Given these data, we conclude that K-Ras may activate PKCε through PLCε protein–protein interactions.

RETRACTED

**Figure 4:** The PLCε, PKCε signaling pathway is regulated by K-RAS. **(A)** Lentivirus-shK-Ras inhibited the protein and mRNA expression levels of PLCε and PKCε in CRPC cells. **(B)** Activated K-Ras mutant K-RasG12C mRNA expression level of K-RasG12C **(C)** Expression of PLCε and PKCε in R-Bica cells and R-B+D cells detected by Western blot and qPCR. Cells were infected with activated K-Ras mutant K-RasG12C or with K-RasG12C combined knockdown of PLCε. **(D)** The expression of PLCε in Membrane and Cytoplasm in R-Bica and R-B+D cells by Western blot. **(E)** Co-IP studies were performed with K-Ras, PLCε, and PKC ε in R-Bica and R-B+D cells. sh, small hairpin; shPLCε, PLCε knockdown. Vector, empty vector of overexpression K-RasG12C lentivirus. NC, negative control for Lentivirus-shPLCε.*P < 0.05, **P < 0.01, ***P < 0.001; ns, no statistical significance.

### Knockdown of K-Ras Can Inhibit Metastasis, Invasion, and Proliferation of CRPC Cells Through PLCε/PKCε

To test whether the expression of PKCε in CRPC cells was related to drug resistance, metastasis, and invasion, CRPC cells were infected with three lentiviral shRNAs specific for PKCε and #3 lentiviral shRNA markedly reduced the mRNA and protein expression of PKCε, and following the expression of metastasis-related factors, they were decreased at the protein and mRNA levels (Figures 5A,B). Additionally, silenced-PKCε suppressed Transwell invasion and wound healing and partly restored drug sensibility (Figures 5C,E). Previously, we verified that K-Ras regulated PKCε through membrane bound PLCε. Thus, we suggested that knockdown of K-Ras suppressed metastasis, invasion, and migration in CRPC cells and partly restored CRPC drug sensitivity through PKCε by attenuation of the expression of PLCε.

RETRACTED

**Figure 5:** K-Ras regulates protein and mRNA factors of invasion and migration via PKCε. **(A)** CRPC cells were infected with sh lentiviral PKCε; Western blotting and qPCR analyzed the expression of PKCε. **(B)**The expression of VEGF, MMP2, and MMP9 in CRPC cells was detected by Western blot and qPCR. **(C,D)** The R-Bica and R-B+D cell metastasis capacities were assessed by the method of Transwell and wound-healing assays. **(E)** The IC_50_ of R-Bica and R-B+D cells following treatments with LV-shPKCε and LV-NC was analyzed by CCK-8 assay. Cells were infected with a negative control or shPKCε or shK-Ras+PKCε. NC, negative control for Lentivirus-shK-Ras and Lentivirus-shPKCε; sh, small hairpin; shK-Ras, K-Ras knockdown; shPKCε, PKCε knockdown. ***P < 0.001.

### Inhibitor 9 Inhibits the Invasion and Migration of CRPC Cells and Partly Restored Drug Sensitivity *in vitro*

Next, we sought to determine the effect of pharmacological inhibition of K-Ras on malignant behavior of CRPC cells. K-RasG12C is the common mutation activating K-Ras, whose inhibitors are scheduled to be put into clinical use in different types of tumor this year; given this, we chose inhibitor 9 as K-RasG12C inhibitor for *in vitro* and *in vivo* evaluation. *In vitro*, we used 5 μM inhibitor-9 as the experimental group. Following treatment, the mRNA and protein expression of metastasis-related factors VEGF, MMP2, and MMP9 was significantly decreased when evaluated by RT-qPCR (Figures 6A,B). Increasing inhibitor 9 concentrations significantly reduced cellular activities and the IC_50_ of CRPC cells showed that inhibitor 9 significantly restored drug sensitivity (Figures 6C,D). Herein, we provide evidence that inhibitor 9 can markedly suppress metastasis of CRPC cells and partly restored CRPC drug sensitivity *in vitro*.

**Figure 6:** Inhibitor 9 regulates protein and mRNA expression of invasion-related factors and partly restored drug sensitivity. **(A,B)** The expression of VEGF, MMP2, and MMP9 in CRPC cells was examined by qPCR and Western blot. **(C)** CRPC cells were incubated with increasing concentrations of inhibitor 9 (5, 10, 20, 30, 40, 60, 80, and 100 μM) or BLANK for 48 h, and cell viability was analyzed by CCK-8 assay. **(D)** R-Bica cells were incubated with increasing concentrations of bicalutamide, while R-B+D cells were incubated with increasing concentrations of bicalutamide and docetaxel for 48 h, and the IC_50_ of R-Bica and R-B+D cells following treatment with inhibitor 9 and BLANK was determined by CCK-8 assay. ***P < 0.001.

RETRACTED

### Inhibitor 9 Combined With Androgen Deprivation Therapy or Chemotherapy Can Partially Restore Drug Sensitivity and Inhibit Invasion and Metastasis in CRPC Cells *in vivo*

We confirmed that inhibitor 9 can act as an inhibitor of K-RasG12C and, when combined with drugs (bicalutamide or bicalutamide and docetaxel), can suppress metastasis of CRPC cells and increase the sensitivity of CRPC cells to drugs *in vitro*. So, we sought to verify these data *in vivo*. Using our nude mouse model, we employed tail vein injection to introduce tumor cells and to evaluate subcutaneous tumor formation and implantation in the left tibia in the bone invasion model. We subjected each to various treatments in order to observe changes in visceral metastasis and bone invasion and drug resistance. In the three animal models, thinking about the drug docetaxel, the dose of either inhibitor 9, chemotherapeutic, or PBS was 10 mg/kg. CRPC cells were given to establish the tumor model. Treatments were then started on the 14th day after CRPC cells were given using a program of 5 days on and 2 days off until 42 days. No mice were sacrificed as a result of reaching pre-established humane endpoints.

As a metastatic animal model, R-Bica cells and R-B+D cells transfected with lentivirus expressing firefly luciferase were injected via the tail vein in our nude mice. We detected tumor metastasis using visualization on an IVIS Lumina II each week. The intensity of fluorescence is expressed by radiance, p/s/cm^2^/sr. Metastasis in nude mice at 21 and 42 days was shown in Figures 7B,C. It can be seen that animals that were not treated with labeled cells had no fluorescence on the live imager (Figure 7A). Meanwhile, HE stain can confirm sections of metastatic tumors in lung (Figure 7A), and in this experiment, we were able to confirm the injection of R-Bica or R-B+D cells into the mice. We were also able to show a marked decrease in metastasis when cells were treated with inhibitor 9. This result indicated that inhibitor 9 combined with drugs could effectively inhibit visceral metastasis of CRPC cells. Next, CRPC cells were injected into the right flank to create the subcutaneous tumor model or treated in the same way as the general metastasis model. Following 42 days of treatment, mice were killed and tumors were excised and then measured (Figure 7E). We were able to conclude that either R-Bica or R-B+D cells groups were treated with inhibitor 9; the tumor volume was significantly decreased when compared to the control group. These results suggested that inhibitor 9 suppressed tumor growth in the CRPC xenografts and partly restored drug sensitivity *in vivo*. In the bone invasion model, the same treatment was undertaken and tumor formation was evaluated using weekly X-ray and finally stained by HE. After 42 days, we concluded that treatment of either R-Bica or R-B+D cells with inhibitor 9 significantly decreased bone invasion when compared to control groups (Figure 7D).

RETRACTED

**Figure 7:** The combination therapy of inhibitor 9 and drugs can partially restore drug sensitivity and inhibit invasion and metastasis in CRPC cells *in vivo*. **(A)** No treatment with labeled cells had no fluorescence and H&E-stained sections of metastatic tumors in lung. T, tumor and L, lung. **(B,C)** The nude mice at 21 and 42 days after tail vein injection with CRPC cells transfected with lentivirus expressing firefly luciferase captured by bioluminescent imaging (signal intensity is represented by radiance, p/s/cm^2^/sr). **(D)** Hematoxylin and eosin staining and X-ray were used to detect the bone invasion of nude mice. **(E)** Tumor sizes and dynamic growth of subcutaneous tumors (***P < 0.001). **(F)** Schematic diagram summarizing our study: Knockdown of K-Ras can inhibit metastasis, invasion, and proliferation and partly restored drug sensitivity through PLCε/PKCε in CRPC cells; inhibitor 9 combined with drugs can down-regulate the expression of K-RasG12C and delay the progression of CRPC.

In summary, our study concluded that inhibitor 9 combined with drugs can inhibit visceral metastasis and bone invasion of CRPC cell lines R-Bica, R-B+D cells, and inhibited the tumor growth and increased drug sensitivity *in vivo*.

## Discussion

Identifying the appropriate treatments for CRPC is challenging due to progression of malignancy. In recent years, articles have reported that point mutations in K-Ras are related to drug resistance, invasion, and metastasis in different types of tumors (25, 46–48). The present study found that the expression of K-Ras in CRPC tissues was higher than that in PPC tissues. Of note is that high expression of K-Ras was correlated with increased metastasis and drug resistance as well as in different CRPC cell lines. More importantly, in CRPC patients, recurrence-free survival was associated with the expression of K-Ras. Thus, the up-regulation of K-Ras gene may be associated with the progression of prostate cancer.

The expression of PKCε has been reported to be reduced in androgen-dependent cells and up-regulated in CRPC cells (28–31). In this study, we also revealed an underlying mechanism that PKCε increase was related to prostate cancer progression, suggesting that PKCε could be used as a marker for prostate cancer recurrence.

RETRACTED

Current reports suggest that K-Ras may play a crucial role in regulating the progression of tumors, such as colon cancer (49) and cholangiocarcinoma (50). In addition, it can also activate multiple signaling pathways and regulate the procession of tumors (51–53). Meanwhile, the present clinical study found that not only the expression of K-Ras, PLCε, and PKCε was elevated in CRPC tissues, but K-Ras was also positively correlated with PLCε and PKCε, respectively. Moreover, due to the unique structure of PLCε, RA domain can directly bind to the genes of K-Ras, and the EF, X, and F domain can activate DAG/CA2^+^ to activate PKCε (37). Therefore, it is suspected that K-Ras may activate PKCε through PLCε. To confirm this hypothesis, drug-resistant cell lines with genetic backgrounds and drug resistance similar to our clinical patients were generated using androgen-dependent LNCaP cells as a base. It is worth noting that we first revealed that K-Ras may bind directly to PLCε and that PLCε may bind directly to PKCε via protein–protein interactions to regulate metastasis and drug sensitivity of CRPC cells. Additionally, we first demonstrated that K-Ras modulated PKCε through regulating the expression of PLCε in the membrane in CRPC cells. However, membrane targeting may not be the only reason for PLCε-mediated up-regulation of PKCε in CRPC cells.

Some studies reported that the main reason for the activated K-Ras was the mutation of K-RAS and the common mutation of K-Ras was K-RASG12C [21]. Therefore, a K-RasG12C inhibitor (inhibitor 9), which was similar to new clinical drugs, was used for different types of tumors, which can irreversibly bind to K-Ras mutants (20). The experiment results were obtained similar to those in our knock-down studies *in vitro*. The correlation between K-RasG12C expression, visceral metastasis, bone invasion, and drug resistance of CRPC cells was then verified. Here, our data showed that administration of inhibitor 9 combined with drugs (bicalutamide or bicalutamide and docetaxel) could suppress metastasis and invasion of CRPC cells and partly restore drug sensitivity *in vivo*. These results confirm the value of this type of drug in the treatment of K-Ras-associated castration-resistant prostate cancer.

To the best of our knowledge, this study first explored that K-Ras may bind directly to PLCε and that PLCε binds directly to PKCε through protein–protein interactions. These interactions enhance metastasis and reduce drug sensitivity of CRPC cells. The oral inhibitor of K-RasG12C has entered the clinical trial and is expected to be an ideal treatment for castration-resistant prostate cancer (Figure 7F).

RETRACTED

## Data Availability Statement

All data generated or analyzed during this study are included in this article.

## Ethics Statement

The studies involving human participants were reviewed and approved by the Ethics Committee of Chongqing Medical University. The patients/participants provided their written informed consent to participate in this study. The animal study was reviewed and approved by the Ethics Committee of Chongqing Medical University. Written informed consent was obtained from the individual(s) for the publication of any potentially identifiable images or data included in this article.

## Author Contributions

JL, XW, and YG designed the experiments. YZ, YG, ZQ, LL, XW, and CL collected the specimens and analyzed the clinical data. JL, YG, TL, LD, and JY carried out the experiments. JL wrote the manuscript. ZQ, CL, and XW provided technical support of this research project and supervised the progress of the experiments. JL, YZ, and YG analyzed the statistical data. JL, LL, TL, and BQ assembled and installed the figures. All authors have read and approved the final manuscript.

### Conflict of Interest

The authors declare that the research was conducted in the absence of any commercial or financial relationships that could be construed as a potential conflict of interest.
